RETRACTED

# Application and Prospect Analysis of Artificial Intelligence in the Field of Physical Education

**DOI:** 10.1155/2022/1042533

**Published:** 2022-08-13

**Authors:** Wujun Xiang

**Affiliations:** School of Physical Education, Jianghan University, Wuhan 430056, Hubei, China

## Abstract

The development of AI technology has a significant impact on every sector of business. Artificial intelligence uses this technology to reduce the amount of work required, duplicate work, and increase the accuracy of work by modelling human behaviour and thought. On the basis of a thorough analysis of artificial intelligence technology, the technology is applied to teaching, specialised training, and specialised testing in response to the current issues in the field of physical education and the business that can be improved through auxiliary tools. The paper discusses how artificial intelligence technology can be used in physical education. After that, it examines how physical education is currently taught in classrooms and discusses how artificial intelligence is affecting this field. Following a thorough demonstration of the aforementioned material, the commonly used artificial intelligence technologies are introduced in turn, along with the methodology used in physical education. The use of computer models in physical education is then explained, and future analysis is conducted on the basis of this information.

## 1. Introduction

Artificial intelligence, which can simulate, extend, and expand human intelligence, is a field of study built on the foundations of many other fields, including computer science, cybernetics, information theory, systems science, and philosophy. In essence, computer science has a subfield called artificial intelligence. The public generally accepts the quick development of computer application technology because it exhibits greater intelligence and applicability. Due to the country's top-notch design and effective artificial intelligence policies, the characteristics of artificial intelligence application and physical training education are more closely related and support one another. The rapid development of artificial intelligence is an indispensable backbone in the process of accelerating the modernization of education benefit. The data support of artificial intelligence in education and teaching has grown steadily stronger with the advancement of Internet of Things technology. More thorough scenarios are provided, along with novel application scenarios. Machine learning is now the primary artificial intelligence research area and application paradigm. Intelligent processing is based on precise data processing and is taught through data training sets. An unavoidable trend in modern development is the advancement of artificial intelligence in subject education, and this trend will significantly advance school sports reform and development [1, 2].

RETRACTED

## 2. The Application of Artificial Intelligence in Sports

There are numerous ways to categorise sports. This paper divides sports into three categories based on their use as application objects for artificial intelligence: competitive sports, school sports, and mass sports. The application status of AI in these three categories of sports is briefly described as follows.

### 2.1. The Application of Artificial Intelligence in Competitive Sports

Competitive sports require high accuracy, and in the process of competition, both parties need to follow certain sports rules to complete. It is characterized by sports competitions and is a social sports activity with the main goal of giving full play to the spirit of sports competition based on sports rules. At present, artificial intelligence [3, 4] is widely used in competitive sports and has penetrated into all aspects of competitive sports, such as athlete quality testing, competitive sports training, action analysis and tactical modelling, auxiliary referees, and intelligent referees.

### 2.2. The Application of Artificial Intelligence in Mass Sports

With the continuous integration of artificial intelligence and the sports and fitness market, a large number of intelligent fitness products have gradually entered the consumer market. Wearable smart devices such as smart bracelets and smart sports shoes are gradually appearing in people's daily fitness. With the rapid update and iteration of smart products entering the consumer market, the integration of AI and mass fitness has been accelerated.

### 2.3. The Application of Artificial Intelligence in School Sports

At present, the application [5, 6] of artificial intelligence in the field of school sports is still in its infancy. For example, universities enable intelligent venues to efficient data and optimize business processes, save time, and improve services; intelligent physical fitness testing systems can be applied to students' physical fitness testing files, exercise risk prediction, training on new scientific fitness methods, and fitness effect monitoring. These practical explorations have opened a useful beginning for the field of artificial intelligence-enabled school physical education.

## 3. Current Situation of Physical Education in Schools

It is an indisputable fact that the quality of school physical education is not high and the teaching efficiency is low. Teachers can only rely on personal experience and cognition to carry out teaching. The teaching design, content setting, and adjustment lack an effective scientific basis, and there is a trend of random teaching. The effect of physical education is limited by many shortcomings. For example, teachers' explanation and demonstration are limited by the influence of skill level, physical quality, and age, and the demonstration effect is difficult to guarantee. Teachers do not understand the specific needs of students and the basics of physical education and carry out unified progress teaching. Students learn in confusion and passive indoctrination, resulting in students' physical problems such as poor physical learning atmosphere and strong resistance.

RETRACTED

## 4. The Main Technical Path for Artificial Intelligence to Empower School Physical Education

The combination of artificial intelligence and physical education is a new trend in contemporary school physical education [7]. According to the iterative development of equipment and technology, the main technical paths for artificial intelligence to empower school sports are intelligent wearable devices, sports vision technology, and intelligent sports venues and VR etc.

### 4.1. Smart Wearables and School Sports

Smart wearables may be advertised as jewellery, watches, clothing, or other accessories. It makes use of contemporary communications and sensors to record a range of bodily life data and track the health of the human body. Basic characteristics of wearable artificial intelligence products include portability, pertinence, real-time, and safety [8]. Smart clothing can monitor a wide range of physiological parameters, including electromyography, respiration, body temperature, heart rate, blood pressure, blood oxygen saturation, blood sugar, and other physiological indicators, in both active and passive students. Motion sensors are demonstrating the continued development of deep intelligence, diversification, flexibility, and wearability as a result of technological update and iteration, multifunctional device integration, big data analysis and processing, and other technologies. These technologies can conduct thorough and thorough analyses of the signals produced during the process of sports training. Sports big data of sports trainers are built using multiangle and multilevel mining. Smart wearable devices used in physical education can assist teachers in quickly assessing students' exercise load and other physiological indicators, which is crucial for preventing sports-related injuries and scientifically regulating teacher behaviour. Smart wearables also foster a more balanced understanding of sports among students and help them realise the multilevel empowerment impact of smart technology on physical education in schools.

RETRACTED

### 4.2. Sports Vision Technology and School Physical Education

The application of sports vision technology in physical education can accurately and intelligently identify the actions of students [9] and solve the practical dilemma that teachers cannot take into account the students' simultaneous learning and practice. The application of computer vision technology can help students clearly understand the gap between their own technical movements and standard movements in terms of completion quality, amplitude, angle, movement trajectory, etc. Changes in know-how. The application of computer vision technology not only deepens students' cognition of movements. At the same time, it can mobilize the training interests of trainers.

### 4.3. VR and School Physical Education

VR is a computer simulation system that can create and experience virtual worlds, and users can get the most realistic feeling in the illusory world. The huge potential is shown by VR technology. With the maturity of technology, it has been successfully applied in the field of competitive sports and achieved good results. With the advent of the VR era, it makes the traditional school physical education ideas, plans, and methods have a greater impact and also provides better opportunities for physical education improvement. The application of VR technology in physical education can change the traditional teaching and learning methods, solve the problems of poor teacher's explanation and demonstration effect, lack of situational guidance and students' difficulty in imitating and understanding under the traditional teaching mode, so that students can obtain the experience close to the real situation [10, 11]. The three-dimensional and immersive action experience can be simulated and practiced in the set VR situation, helping students to practice better, faster, and more interestingly.

## 5. The Impact of Artificial Intelligence in School Sports

Artificial intelligence empowers school physical education, which can bring beneficial changes and positive effects to teachers' teaching mode, student learning mode, teacher's teaching evaluation, student learning evaluation, and student learning effect.

### 5.1. The Impact of Artificial Intelligence-Enabled Physical Education on Teaching Mode

Clarifying teaching objectives, explaining and demonstrating concepts, and guiding and summarising learning activities are all part of the traditional physical education teaching process. The core of the physical education teaching method is comprised of the teacher's explanation, demonstration, and practise guidance. The influence of skill level, physical quality, and age limits the impact of a teacher's action demonstration. It can be challenging to ensure that students are learning something new because teachers frequently find it difficult to teach complex movements through demonstrations and must instead rely solely on their own explanations [12]. In addition, it can be challenging for teachers to explain and demonstrate some complex skill movements, especially when doing so slowly from multiple angles. This makes it difficult for students to comprehend and imitate what is being demonstrated, which has a negative impact on learning popular. In order to help students better understand the internal logical relationships between sports actions and develop deep-level skill cognition, VR artificial intelligence technology can simulate real sports scenes and slowly show the details of sports from various angles. In terms of practise guidance, teachers frequently have to direct the majority of students to practise at the same time, making it difficult for them to identify each student's movement practise in time. This may cause some students to practise repeatedly with incorrect movements, resulting in movements that are challenging to correct stereotypes. With the aid of computer vision technology and related intelligent algorithms, teachers are better able to identify incorrect student practise behaviours and correct them quickly. In order to fully comprehend their own actions and those of others, students can also use computer vision technology's playback and action comparison features. variations in accepted practises. The development of a highly effective and precise physical education teaching method is strongly supported by the advancement of AI technology.

RETRACTED

### 5.2. The Impact of Artificial Intelligence-Enabled Physical Education on Students' Learning Patterns

Traditional physical education classes do not engage students because they do not feel like themselves. The fact that teachers are unable to provide students with individualised instruction based on their unique foundations and receptive abilities is one of the key contributing factors. Students learn in confusion and lack motivation because teachers lack a clear understanding of the fundamentals of physical education and the needs of individual students. A new avenue for students' physical education learning is opened up by the integration of artificial intelligence technologies like sports vision, smart wearables, and VR. Utilizing wearable technology, virtual reality (VR) technology can gather knowledge from students and acquire real-time, multiperspective image information. It is possible to provide detailed evaluation and information on the three-dimensional motion. To help teachers carry out targeted teaching design and guidance so that students can transition from a unified learning mode to a personalised learning mode, artificial intelligence technology enables big data of students' movement to be obtained in real time and the quality of movement to be fed back in real time. The interaction between teachers and students can be carried out effectively with the help of artificial intelligence, and students can now learn in a personalised way, which has a significant positive impact on their motivation and interest [13].

RETRACTED

### 5.3. The Impact of Artificial Intelligence-Enabled Physical Education on Student Learning Evaluation

An efficient way to raise the standard of physical education instruction is to evaluate the teaching abilities of teachers. The two main aspects at the moment are student evaluation and supervision evaluation. There are some issues with the supervision evaluation, such as the evaluation's single subject, subjective results, flashy content, and failure to demonstrate the improvement's goal [14], which has little bearing on the teaching of physical education's quality. Students should receive objective evaluations because they are involved directly in the teaching process, but this is not the case. Most students rate teachers on a good or bad scale, depending on factors like how strict the discipline is, how much time is spent resting, and other factors. Under the influence and change of artificial intelligence technology, information about students' effective exercise time, exercise physiological load, and movement completion quality can be quickly gathered. Big data can be mined and analysed to reveal whether or not teachers' lesson plans are sensible and whether or not students are learning anything. A key factor in determining how well it meets the standard is the teacher's teaching evaluation. A new avenue for the reform of the current teacher evaluation system has been made possible by the mining and analysis of big data.

### 5.4. The Impact of Artificial Intelligence-Enabled Physical Education on Teaching Evaluation

At present, teachers' evaluation of students' learning mainly includes process evaluation and summative evaluation. Summative evaluation is the examination evaluation, which has specific and quantifiable evaluation indicators [15, 16],. The process evaluation is composed of attendance and classroom performance, in which classroom performance is the main content. Class performance is mainly to evaluate the seriousness of students' learning. To measure the seriousness requires not only qualitative subjective evaluation, but also quantitative objective evaluation, and the two complement each other. In traditional physical education teaching, it is difficult to obtain and accurately count the sports big data indicators such as exercise time, exercise load, maximum heartbeat, and average heartbeat. This makes the fairness and objectivity of the process evaluation questionable and weakens the promotion effect of the process evaluation on students' physical education learning. Under the empowerment of artificial intelligence technologies such as sports vision, flexible smart wearable devices and intelligent big data analysis, students' sports data indicators can be easily obtained, which provides effective technology for the development of quantitative evaluation and improves the teaching process. The accuracy of sexual evaluation improves the objectivity and scientificity of teachers' evaluation of students' learning as a whole.

RETRACTED

## 6. Artificial Intelligence Technology Commonly Used in the Field of Physical Education

Artificial intelligence models and algorithms are used in physical education work. The commonly used machine learning models [17] are described as follows.

### 6.1. Convolutional Neural Network

The traditional neural network achieves feature extraction through multiple activation function compounding, splicing, layering, and other steps. The automatic learning of the network reduces the workload of manual feature extraction, but the feature model extracted by the traditional neural network is one-dimensional, which is not suitable for some. Features that are spatial in nature are very disruptive. For this reason, scholars have proposed Convolutional Neural Networks (CNNs). In recent years, CNN has become a hot spot for scholars to study artificial intelligence, and it is mostly used in the standardized monitoring of sports training movements.

In the course of physical education, mistakes are frequently made during the movement process after students learn the movements for the first time because the connection between the nerves and muscles of the main body of the movement is not yet precise. Physical education teachers must therefore learn how to correct and prevent incorrect movements in order to enhance the quality of their instruction in sports technology. According to pertinent research and investigation, in the past, it was difficult to accurately identify incorrect movements during physical education training, which made it difficult to correct them in a timely manner. Therefore, the convolutional neural network can be used as the basis for improving the wrong action detection process in physical education training through deep learning by adding a batch normalisation layer in the middle of the convolution layer and the pooling layer. This will address the aforementioned shortcomings. Standardize incorrect action samples from physical education training in batches, extract incorrect action features from these, quickly and precisely identify incorrect actions from physical education training, and raise athletes' sporting proficiency.

RETRACTED

The specific network model structure is shown in Figure 1.

The calculation formula of the output of the convolutional layer is shown in the following equation:

(1) $$\begin{array}{c} y_{j}^{m}=\sum_{i}x_{i}^{m-1}\times k_{ij}^{m-1}+b_{j}^{m}. \end{array}$$

Here, *y*_*j*_^*m*^ represents the output value of the *j*-th unit in the *m*-th layer of the convolutional layer, *x*_*i*_^*m*−1^ is the *i*-th matrix input in the *m* − 1 th layer in the layer, *k*_*ij*_^*m*−1^ is the convolution kernel that connects the input *i*-th matrix and the *j*-th unit between the *m*-th and *m* − 1 layers in the convolutional layer; *b*_*j*_^*m*^ is the feature map output by the *m*-th layer. Bias value for *j* cells. The feature matrix calculated by formula (1) in the convolution layer can be processed by a nonlinear activation function and converted into a corresponding high-order matrix to enhance the nonlinear expression ability of the CNN network model.

Equation (2) is the full connection output calculation formula.

(2) $$\begin{array}{c} y_{j}^{m}=\underset{i}{\sum }w_{ij}^{m-1}\times x_{i}^{m-1}+b_{j}^{m}. \end{array}$$

Here, *y*_*j*_^*m*^ represents the output result of the *j*-th unit in the *m*-th layer of the fully connected layer, and *w*_*i*_^*m*−1^ is the *i*-th unit and the *m*-th unit in the *m* − 1-th layer of the fully connected layer. The weight value of the conversion between *j* units in the layer, *x*_*i*_^*m*−1^ is the value of the *i*-th unit in the *m* − 1th layer in the fully connected layer, and *b*_*j*_^*m*^ is the *j*-th unit in the *m*-th layer offset value. After calculating the output feature matrix, normalize each element of the matrix, limit the value between 0 and 1, and each element sums to 1, and the category represented by the maximum value is the category to which the sample belongs.

In order to prevent overfitting due to the small scale of the dataset used in the process of deep convolutional neural networks, a regularization method is often introduced in the fully connected layer. The network structures corresponding to the data sets are not consistent, but all network weights are shared, which can greatly improve the stability of the wrong action detection model for physical education training and make it less complicated for each neuron to adapt to each other.

RETRACTED

The depth of the neural network determines the improvement in the accuracy of wrong action detection during sports training, and features have a positive correlation with representational capacity. The wrong action data's features will all be calculated by the deep neural network, and the more features are extracted, the deeper the final output the greater the aptitude. The phenomenon of gradient disappearance is easily experienced during the process of increasing network depth, which lowers network performance. ResNet101, which can extract the subtle features of the physical education training sample data faster and better in the middle of the convolution layer and pooling layer, is the basic network used to extract features using deep convolutional neural networks to solve this problem. The data transmission strategy is modified while the network training speed is accelerated, and further network performance optimization is encouraged by adding a normalised layer and residual blocks in batches of ResNet.

### 6.2. Recurrent Neural Network

Recurrent Neural Network (RNN) [18, 19] takes sequence data as the input of the model, and the output of each layer in the model can be used as part of the information content as the input of the next layer. Therefore, RNN has the characteristics of memory context, and it has the characteristics of memory context. And, the semantics covered are more sensitive, so RNN can be widely used in text information, natural language processing, and other fields. The output results of RNN are influenced by the previous learning content, so the output results at a particular time may incorporate the features learned from prior learning. RNN can accept irregular sequence data items that are not specified in advance. In the hidden layer of the CNN model, the previously discovered eigenvalues are stored as vectors. One or more output sequences can be produced from one or more input sequences from the standpoint of the input and output structure, and even when the input conditions are the same, the output results may differ.  Figure 2 shows the structure of the RNN model.

Figure 2 describes the RNN model structure, where *W* represents the weight value from *x*_*t*_ to *h*_*t*_, *U* represents the weight value between the hidden layers *h*_*t*−1_ and *h*_*t*_, and *V* represents the weight value from *h*_*t*_ to the output *y*_*t*_. *x*_*t*_ represents the input training sample of the *t*-th layer; *h*_*t*_ represents the hidden feature of the *t*-th layer, and its value is calculated by *x*_*t*_ and h_*t*−1_; *y*_*t*_ represents the output of the *t*-th layer, which is only determined by *ht*. The calculation formula of the RNN model is shown in (3) and (4).

(3) $$\begin{array}{c} h_{t}=f\left(Wx_{t}+Uh_{t-1}\right), \end{array}$$

(4) $$\begin{array}{c} y_{t}=g\left(Vh_{t}\right). \end{array}$$

Equation (3) represents the vector output calculation in the hidden layer of the RNN model, and equation (4) represents the calculation of the output result.

RETRACTED

### 6.3. Long Short Term Memory Network

The CNN model described above has the property of context memory, but when CNN processes long sequence data, it uses backpropagation to transfer the gradient of this layer to the previous sequence, so CNN cannot memorize long texts and is not suitable for some Long sequence data processing work. To solve this problem, with the continuous improvement of CNN, some improved models have been gradually proposed, of which Long Short-Term Memory (LSTM) is the most widely recognized network.

LSTM is regarded as a variant of a more advanced CNN network, which consists of 5 main parts.  Figure 3 shows the LSTM model structure diagram.

1. Unit state: indicates the internal memory information of the network unit
2. Hidden state: the external hidden state acts on the prediction results of the model calculation
3. Input gate: determine which external all inputs can currently be sent to the unit state
4. Forgetting gate: in the previous unit state, decide which ones can be sent as input to the current unit state
5. Output gate: in the current state, decide which units can be input to the hidden state

In the LSTM model, the current unit state is affected by two aspects: one is dependent on the input in the current state, and the other is dependent on the previous unit state, so the LSTM can perform each element in the unit state at a certain moment. Update or forget processing, forming a stable state-dependent mechanism.

In the LSTM model, the unit state calculation of the forget gate is calculated by the following equation:

(5) $$\begin{array}{c} f_{t}=\sigma \left(\omega_{f}•{\left[h_{t-1},x_{t}\right]}^{T}+b_{f}\right). \end{array}$$

Here, *ft* is the information lost by the forget gate at time *t*, *ht* − 1 is the output state of the hidden layer at time *t* − 1, *xt* is the current input, [*ht* − 1, *xt*]*T* is *ht* − 1 and *xt A* matrix is formed, which is multiplied by the weight matrix *ωf*, and then added with *bf*, (*bf* is the bias matrix).

Then, *ct* can be calculated, and its calculation formula is

(6) $$\begin{array}{c} c_{t}=f_{t}c_{t-1}+i_{t}{\tilde{c}}_{t}, \end{array}$$

Here, *c*_*t*_ is the current unit state at time *t*, and c_*t*−1_ is the unit state at time *t* − 1. ${\tilde{c}}_{t}$ is the updated state of the cell, it is the information that the input state is saved to the unit, where it is represented by equation (7) and *c*_*t*_ is represented by equation (8).

(7) $$\begin{array}{c} i_{t}=\sigma \left(\omega •{\left[h_{t-1},x_{t}\right]}^{T}+b_{i}\right), \end{array}$$

(8) $$\begin{array}{c} {\tilde{c}}_{t}=\tanh\left(\omega_{c}•{\left[h_{t-1}\right]}^{T}+b_{c}\right). \end{array}$$

In equations (7) and (8), *b*_*i*_ and *b*_*c*_ are bias matrices. *ω* and *ω*_*c*_ are weight matrices. *σ* is the activation function used.

RETRACTED

LSTM can obtain the features of past time series information. In some processing work, future time series information features are required, so a Bi-LSTM model composed of forward LSTM and post LSTM is proposed. The Bi-LSTM model is shown in Figure 4.

### 6.4. Gate Recurrent Unit

Due to the shortcomings of RNN in the model calculation, such as many parameters, long training time, and complex calculation, in order to improve the processing efficiency of the model, scholars have proposed a simpler model GRU (Gated Recurrent Unit) [20] on the basis of LSTM. GRU combines The unit state and hidden layer state of LSTM to replace the forget gate and input gate of LSTM with the update gate. GRU consists of an update gate and reset gate. Its model realizes the function of LSTM, but its parameters are more refined and its structure is simpler.  Figure 5 is a structural diagram of the GRU model.

In the whole model, GRU uses a reset gate and update gate to control information. The reset gate is used to determine the combination of the input *x*_*t*_ at the current moment and the memory information, and the update gate is used to determine the memory content saved above. The reset gate output *r*_*t*_ is calculated as equation (9), the update gate output *z*_t_ is calculated as equation (10), and its inputs are *x*_*t*_ and h_*t*−1_, which are the input at time *t* and the implicit state at time *t* − 1, respectively, $\tilde{h_{t}}$ and *h*_*t*_ calculation formulas are (11) and (12).

(9) $$\begin{array}{c} r_{t}=\sigma \left(W_{r}x_{t}+U_{r}h_{t-1}\right), \end{array}$$

(10) $$\begin{array}{c} z_{t}=\sigma \left(W_{z}x_{t}+U_{z}h_{t-1}\right), \end{array}$$

(11) $$\begin{array}{c} \tilde{h_{t}}=\tanh\left(U_{h}x_{t}+\left(r_{t}⊙h_{t-1}\right)W_{h}\right), \end{array}$$

(12) $$\begin{array}{c} h_{t}=\left(1-z_{t}\right)⊙\tilde{h_{t}}+z_{t}⊙h_{t-1}. \end{array}$$

## 7. Outlook

Physical education is currently at a stage where the use of artificial intelligence technology is typically in its early stages. Both the consumer demand for sports artificial intelligence equipment and the sports database that serves as the foundation for physical education enabled by artificial intelligence are still in their infancy. In addition, there is no established regulatory framework for smart devices. Since physical education is a relatively new field, its fundamental theoretical foundation is still lacking. It is essential to continue promoting the development and advancement of sports artificial intelligence equipment. Develop intelligent equipment and support the deep integration of equipment and physical education. In terms of policy, it is necessary to direct or create pertinent incentive policies and provide corresponding support in line with industrial policies. From a technical standpoint, a physical education mechanism that combines data resource sharing and business model sharing can be established, and through technological innovation, the drawbacks that the general public are concerned about, like the protection of personal data, can be resolved. In order to increase consumer interest in purchasing sports artificial intelligence equipment, it is necessary to increase the marketability and cost-effectiveness of products. Artificial intelligence-based sports equipment is in extremely high demand, particularly in the fields of school sports and public fitness. Market demand serves as a catalyst for advancing industrial chain efficiency and technological advancement. A complete production in the field of physical education may result from the development and improvement of the random intelligence algorithm and model. To achieve the technology empowerment effect, artificial intelligence equipment costs will move in the direction of civilianization and affordability. Long-term challenges include how to successfully integrate artificial intelligence into the field of physical education in schools. Artificial intelligence can now create more network models thanks to machine learning, which is also being used more and more in physical education. People who work in sports should actively adopt new technology. Computer-assisted instruction, action demonstration, and student action monitoring are all new concepts in physical education. Real-world sports training data collection has become more precise and scientific with the aid of Internet of Things technology. Every person who works in physical education should actively investigate how computer and artificial intelligence technology can be applied to all facets of physical education.

RETRACTED

## Figures and Tables

**Figure 1:** CNN network structure model diagram.

**Figure 2:** RNN network structure model diagram.

**Figure 3:** LSTM model diagram.

**Figure 4:** Bi-LSTM model diagram.

**Figure 5:** GRU network structure model diagram.

## Data Availability

The data used to support the findings of this study are included within the article.
